# Intraoperative sonography may reduce the risk of extensor pollicis longus tendon injury during dorsal entry elastic intramedullary nailing of the radius in children

**DOI:** 10.1097/MD.0000000000011167

**Published:** 2018-06-15

**Authors:** Marcell Varga, Nikoletta Gáti, Tamás Kassai, Szilvia Papp, Sándor Pintér

**Affiliations:** a Péterfy Hospital, Department of Pediatric Trauma Surgery, Budapest; b Department of Trauma Surgery, University Of Szeged, Hungary.

**Keywords:** children, dorsal entry elastic nailing, EPL, ESIN, extensor pollicis longus tendon injury, radius fracture

## Abstract

Extensor pollicis longus tendon (EPL) injury is a potential complication of dorsal entry radial elastic nailing technique in children. The aim of this study was to investigate if intraoperative ultrasonographic guidance can reduce the risk of (EPL) injury.

Correlation between sonographic and operative findings were examined first in 6 adult cadavers. Position of Lister's tubercle, EPL, and extraosseal end of the elastic nail were detected by ultrasound imaging during a minimally invasive dorsal entry nailing. Radial slope of Lister's eminence was determined as a safe and easily identifiable entry point for opening the medullary canal. Extraosseal ends of the nails were bended in a slight radial direction and cut immediately beneath the skin in a maximally palmar-flexed wrist position. Cadaveric dissections followed our procedures all correlated with ultrasonographic findings, we have not seen tendon damage, obstruction or friction by the implant's end.

After cadaveric experiments, we began using intraoperative sonography for monitoring elastic nail insertion in pediatric radial fractures.

Between January 2015 and November 2016, 77 pediatric closed diaphyseal radial fractures were operated by dorsal approach ESIN under intraoperative sonographic checking.

Procedures were executed by 2 orthopedic surgeons experienced in ESIN technique with basic musculoskeletal ultrasonographic qualifications.

Sonographic identification of EPL and Lister's tubercle in the transverse view was possible in all cases. Determination of the position of the nail end to EPL was also possible in all cases. Mean distance of the transverse view center of the EPL and nail was 0.49 cm (range 0.3–0.62 cm, SD = 0.66). Based on the sonographic transverse view, the operator decided repositioning the nails by 2 patients.

We have not found EPL injury postoperatively. All patients were followed for at least 12 months after operations. Nails were removed in all children without further complications.

Intraoperative sonography helps determining optimal insertion point and the risk of EPL injury may be reduced during dorsal entry approach.

Although the procedure is relatively easy, authors take note that surgical and sonoanatomic knowledge, basic sonographic skills and experience in the ESIN technique are equally necessary for its successful application. A greater number of cases is necessary to confirm our initial promising experiences.

## 1 Introduction

Flexible intramedullary nailing (ESIN) of displaced and unstable forearm diaphyseal fractures has become the gold standard operative method in children in the past decades.^[1,2]^

Elastic stable intramedullary nailing of the radius can be carried out from 2 entry points. These are the radial (distal radial side proximally from physis) and the dorsal approaches (through Lister's tubercle)^[3]^ (Fig. 1A and B).

**Figure 1:** (A) X-ray of dorsal entry elastic nailing. (B) X-ray of radial entry elastic nailing.

Both approaches have potential complications. Radial entry point can cause a 2.9% rate of transient and 0.3% rate of permanent injury to the superficial branch of the radial nerve whereas dorsal approach can have a 2.6% rate of extensor pollicis longus tendon rupture.^[4]^ Due to the consequences of these complications, recent studies and the original description advocate using the lateral approach.^[3,5,6]^

Considering that lateral entry ESIN technique is disadvantageous in distal radial diaphyseal fractures and radial nerve may be a source of painful neuroma,^[4,7]^ we were searching for safer ways to reduce the risk of the dorsal approach.

We hypothesized that ultrasonographic checking of the EPL and positioning the end of the nail during insertion in a safe zone can reduce the risk of any damage.

## 2 Methods

Approval of the cadaveric and intraoperative diagnostic study was permitted by our Institutional Medical Board in 2014 November. Ethical permission for cadaveric experiments and clinical use of intraoperative sonography was approved by the Ethics Committee of Péterfy Hospital, in 2014, December.

First, we performed cadaveric examinations on six adult humans.

EPL and Lister's tubercle was visualized by high frequency (14–20 MHz) ultrasound imaging.

After sonographic determination of the insertion points, we positioned an elastic nail through Lister's tubercle according to standard dorsal technique. Position of the EPL relative to the elastic nail was examined from transverse and longitudinal planes.

We bent the extraosseal end of the nail in a slight radial direction and cut beneath the skin in a maximally palmar-flexed wrist position.

This was followed by preparation of the area and comparing the sonographic and anatomic findings (Fig. 2).

**Figure 2:** Relation of the end of the nail to the surrounding structures in dorsal approach. (adult cadaveric preparation) ECRL = extensor carpi radialis longus tendon, ECRB =  extensor carpi radialis brevis tendon, LT =  Lister's tubercule.

Cadaveric dissections all correlated with ultrasonographic findings: distance of EPL and nail was median 0.5 cm (range: 4.4–5.2 cm) clinically, and 0.48 cm (range: 0.44–0.5 cm) sonographically. There was no tendon damage, obstruction or friction.

Following our cadaveric experience, we began using intraoperative ultrasound during elastic nailing of pediatric radial fractures.

A written informed consent was obtained from the parents of all patients.

Between January 2015 and November 2016, 77 radial fractures were operated by dorsal entry elastic nailing with ultrasonic guidance. Inclusion criteria were children with closed and displaced radial or forearm fractures which were candidates for operative ESIN technique. We excluded children with closed growth plates, open fractures and comminuted fractures which could not be stabilized by intramedullary nailing. Patients’ age were between 4 and 15 years and had closed and displaced radial or forearm fractures with open growth plates.

We used aseptically isolated high frequency linear probes and sterile gel for the intraoperative technique. First, we determined the insertion point. After skin incision and soft tissue separation, we targeted the radial slope of Lister's tubercle with a sharp Kirschner wire (Fig. 3). After we pressed the wire softly to the bone we checked its position with image intensifier and ultrasound. Medullary canal opening with a sharp awl was also monitored sonographically and an elastic nail of 2 to 2.5 mm diameter was inserted.

**Figure 3:** Sonography -assisted aiming of the radial side of Lister's tubecule with a K-wire.

Operative technique and fracture reduction were made according to standard protocol.^[3]^

After cutting the end of the nail, we rechecked its position relatively to Lister's tubercle.

EPL has been also checked in longitudinal and transverse plane, we analyzed its relation to the extraosseal part of the nail (Figs. 4–6).

**Figure 4:** Transverse intraoperative sonographic view of the nail and tendon. ESIN = elastic stable intramedullary nail, EPL = extensor pollicis longus tendon, LT = Lister's tubercule.

**Figure 5:** Longitudinal intraoperative sonographic view of the nail and the radius: Extensor pollicis longus tendon is not visualized.

**Figure 6:** Longitudinal intraoperative sonographic view of the radius and the EPL tendon. Nail is not visualized in this plane. EPL = extensor pollicis longus.

Continuity of the tendon has been checked by dynamic examination while passively flexing and extending the wrist and the thumb.

In patients where we found that the nail was too close to the tendon or the EPL got stock during dynamic assessment), we corrected its position.

Procedures were executed by 2 orthopedic surgeons experienced in ESIN technique and with musculoskeletal ultrasonographic qualifications.

## 3 Results

Ultrasonographic identification of EPL and Lister's tubercle in the transverse view was possible in all children.

Determination of the position of the nail to EPL was also possible in all patients. Mean sonographically measured distance of the transverse view center of the EPL and nail was 0.49 cm (range: 0.3–0.62 cm, SD = 0.66) (Fig. 7).

**Figure 7:** Measurement of the distance of the nail and the tendon in transverse sonographic view. LT = Lister's tubercule, EPL = extensor pollicis longus tendon.

Longitudinal view of EPL was not clearly defined in 2 cases.

Based on the sonographic transverse view (insertion points were 2 close (< 0.3 cm) to EPL) the operator decided repositioning the nails by 2 patients.

On one occasion EPL movement was not seen with dynamic assessment, although the tendon was clearly identifiable. In this case, we decided re-bending the end of the nail. After correction, we were able to identify normal tendon movement.

Sonographic procedures took average 5 minutes (range: 2–8 min. mean = 4.8 min) extra time during operations.

We have not found EPL injury or septic complications postoperatively. All patients were followed for at least 12 months after operation. Nails were removed in all children without further complications.

## 4 Discussion

Among the muscles involved in thumb movement, the extensor pollicis longus (EPL) tendon of the hand is considered the most consistent structure with the least variation among individuals.^[8]^ Lister's tubercle is a prominent and sonographically easily visible landmark in the dorsal side of the radius.^[9]^

Intra- and postoperative usage of high-frequency ultrasound in musculoskeletal trauma is a relatively new method for various purposes.^[10,11]^ Recently, few authors have reported good initial results with sonography in different musculoskeletal operations.^[12,13]^

Using sonography is advantageous due to the visualization of the relationship of various soft tissues (i.e. tendons, nerves, arteries) and implants which are invisible to x-rays, and the lack of radiation.^[10–13]^ Ultrasound is also a reproducible tool for identification of EPL and its pathologies.^[9]^

The exact etiology of pediatric EPLT injury in forearm fractures is still a question of debate.

In adult populations direct injury, increased pressure in the third extensor compartment, poor vascularization, chronic mechanical irritation caused by an implant, callus formation or spontaneous idiopathic rupture may be considered as pathogenic factor theoretically.^[14–17]^ Although, there may be other causes,^[18,19]^ since most of the pediatric EPL injuries found in the literature are related to dorsal entry elastic nailing, it seems to be a unique complication of the dorsal approach.^[20–23]^

A small cohort study identified no significant patient characteristics as any predictor of EPL rupture.^[20]^ In a study of 9 pediatric ruptures the nail entry site was directly related to the location of EPL.^[5]^ Direct injury of the tendon during insertion, or chronic irritation caused by the end of the nail can lead to tendon rupture.^[23]^

In a six years period in our institution (between 2010 and 2016) we have performed 354 dorsal entry radial nailing procedures and found 7 EPLT injuries retrospectively. Four cases were identified as acute (<one week after surgery) 3 as chronic (>one week postoperatively) injury. During reoperation, we found 6 complete ruptures. In all chronic and in one acute case extensor indicis tendon transfer has been performed. Direct repair was possible in 2 acute cases. In one case rupture of the EPL tendon was not confirmed intraoperatively: the tendon was mechanically obstructed by the nail, and this caused the block of motion. The reposition of the implant has solved the problem. We hypothesize that a late rupture would have occurred without our early intervention.

Cutting and bending the nail under the skin and above the level of the tendon helps to reduce the risk of skin irritation.^[24]^ Reviewing the literature and our experiences we came to the conclusion that optimisation of the insertion point and the position of the extraosseal end of the nails can reduce the risk of both acute and chronic ruptures. Intraoperative ultrasound has been proven an easy and useful tool for visualizing these optimal reference points. We found that exact sonographic differentiation of Lister's eminence and transverse view of EPLT were easily feasible. The visualization of the end of the nail, and the determination of its position to Lister's eminence and tendon during insertion is more difficult and technically demanding. In spite of this latter fact using sonographic guidance took an average extra 5 minutes during operations. Two times the longitudinal views of tendons were not clearly identifiable. We think this was rather a technical problem in the early learning curve period.

Although the procedure seems very easy, the authors take note that surgical and sonoanatomic knowledge, sonographic skills, and experience in the ESIN technique are equally necessary for its successful application.

## 5 Conclusion

We came to the conclusion that intraoperative sonography may reduce the risk of the dorsal entry ESIN technique. The method is simple, harmless and only slightly increases the surgical time.

A greater number of cases is necessary to confirm our initial promising experiences.

## Author contributions

**Conceptualization:** Marcell Varga, Sándor Pintér.

**Data curation:** Szilvia Papp.

**Investigation:** Marcell Varga, Nikoletta Gáti, Tamás Kassai, Szilvia Papp.

**Methodology:** Marcell Varga.

**Project administration:** Marcell Varga.

**Resources:** Marcell Varga.

**Supervision:** Sándor Pintér.

**Writing – original draft:** Marcell Varga.

**Writing – review & editing:** Marcell Varga.
